This article has been retracted.

# Target Tracking Algorithm for Table Tennis Using Machine Vision

**DOI:** 10.1155/2021/9961978

**Published:** 2021-05-13

**Authors:** Hongtu Zhao, Fu Hao

**Affiliations:** ^1^Physical Education Institute, Jilin Normal University, Siping 136000, Jilin, China; ^2^Jilin Provincial Neuropsychiatric Hospital, Siping 136000, Jilin, China

## Abstract

The current table tennis robot system has two common problems. One is the table tennis ball speed, which moves fast, and it is difficult for the robot to react in a short time. The second is that the robot cannot recognize the type of the ball's movement, i.e., rotation, top rotation, no rotation, wait, etc. It is impossible to judge whether the ball is rotating and the direction of rotation, resulting in a single return strategy of the robot with poor adaptability. In this paper, these problems are solved by proposing a target trajectory tracking algorithm for table tennis using machine vision combined with Scaled Conjugate Gradient (SCG). Real human-machine game's data are obtained in the proposed algorithm by extracting ten continuous position information and speed information frames for feature selection. These features are used as input data for the deep neural network and then are normalized to create a deep neural network algorithm model. The model is trained by the position information of the successive 20 frames. During the initial sets of experiments, we found the shortcomings of the original SCG algorithm. By setting the accuracy threshold and offline learning of historical data and saving the hidden layer weight matrix, the SCG algorithm was improved. Finally, experiments verify the improved algorithm's feasibility and applicability and show that the proposed algorithm is more suitable for table tennis robots.

## 1. Introduction

A table tennis robot [1] refers to a typical real-time intelligent robot playing table tennis with humans. It perceives the service route and trajectory of competitive objects, makes reasonable judgments and return strategies, and achieves flexible hitting. The research of table tennis robot systems involves an extensive range of fields. It integrates knowledge in different areas such as computer vision [2], artificial intelligence [3], automatic control [4], robot kinematics [5], and computer graphics. It has exceptional research value and broad application prospects.

In table tennis, table tennis is small and the flying speed is fast, and it requires table tennis robots to have continuous and rapid response capabilities. It needs to predict the high-speed table tennis trajectory in a short time and make accurate hits. It requires significant efforts to put forward a real-time and precise table tennis robot control. Therefore, table tennis robots' development and broad application need to ensure effective table tennis trajectory prediction [6]. Only under the premise of sufficient analysis of the ball's characteristics, the table tennis robot returns a more timely and accurate action. At present, there is insufficient research on trajectory prediction and a lack of research on spin trajectory recognition. As a result, the research on table tennis robots needs to be further explored. Our study aims to improve the robot's reaction speed, reduce the reaction time, and continue to develop in terms of distinguishing different types of incoming balls based on ensuring the accuracy of returning balls [7].

There are some problems in the current research on table tennis robots. First of all, table tennis is a high-speed moving object, with an average speed of 30 m/s. However, in the existing research, once the speed of the sphere exceeds 10 m/s, it is difficult for the robot to make a correct response in a short time. The second point is that the existing system still cannot judge for different types of incoming balls, for example, up and down spin, left and right spin, etc. The types of incoming balls that can be returned are limited, and the return strategy is single [8].

Based on current research, most of the table tennis robot researchers' work is focused on analyzing the ball's trajectory without spinning. A large amount of trajectory prediction work is also carried out around this object. The shelving of the spin problem is a lack of understanding of the spin motion process. Therefore, this paper takes the table tennis robot as the research background and proposes a table tennis target trajectory and tracking algorithm using deep learning.

The main contributions of this paper are as follows.

1. The sine of the current table tennis robot system cannot determine whether the ball is rotating. The direction of rotation causes the robot's single return strategy and poor resilience. This paper proposes a novel target trajectory and tracking algorithm for table tennis using deep learning. It enhances the predictive ability of the robot system on the trajectory of table tennis.
2. The proposed algorithm is based on the transfer learning theory in deep learning. It uses a layered noise reduction autoencoder to learn a general hierarchical image feature description. The learning process is offline from many auxiliary data in an unsupervised manner through fine-tuning training to model and characterize trajectory characteristics of various tracking targets.
3. The simulation experiments are carried out. The experimental results show that the algorithm in this paper can effectively improve the table tennis robot system's ball returnability and improve the quality of man-machine sparring training.

The rest of the paper is organized as follows. In Section 2, related work is studied, and methodology is given in Section 3. The experimental results are shown in Section 4, and Section 5 concludes the paper.

## 2. Related Work

In the 1980s, research on table tennis robots started abroad. The first table tennis robot developed was just a table tennis ball machine [9]. This kind of robot can only serve but does not have the ability to fight back. It was not until later that it gradually developed into a new generation of table tennis robots that can return the opponent's ball. In 1983, Professor John Billingsley of Portsmouth Polytechnic University in the United Kingdom initiated a robot-playing table tennis competition. From 1985 to 1988, the robot table tennis competition was successfully held four times in Europe in the past four years. The participants were from universities in the United Kingdom, Finland, Sweden, and Switzerland [10]. These competitions have extensively promoted the technical field of table tennis robots. John Billingsley formulated appropriate rules for the robot table tennis game based on optical measurement technology to improve the table tennis robot's success rate returning the ball. The regulation stipulates that the ping-pong table is 2.0 × 0.5 m, which is smaller than the standard size of the ping-pong table 2.7 × 1.5 m, and the space for hitting the ball is limited to three wireframes installed at both ends of the table and on the surface of the net. The ball's trajectory hit by the table tennis robot must pass through these three 0.5 × 0.5 m wireframes, and the opposite robot only needs to move the racket within the metal frame in front of itself to intercept the ball. The table is shown in Figure 1.

In the late 1980s, the Swiss Federal Institute of Technology Zurich designed a six-degree-of-freedom table tennis robot to participate in the international table tennis robot competition [11]. The proposed designed consists of a three-degree-of-freedom mechanical wrist and a three-degree-of-freedom mechanical arm. It uses the parallel distributed computer network of the MC series processor produced by Motorola to complete the measurement, prediction, and control of the robot's trajectory of table tennis. The table tennis robot participated in the table tennis robot competition in Hong Kong and eventually won first place in the event [12].

In 2002, the Miyazaki Laboratory of Osaka University in Japan proposed a method to control a table tennis robot, which can hit the ball to the desired position within a specified time [13]. The proposed system has two rotations and two translation joints, a total of four degrees of freedom. Two motors near the racket control the racket's attitude, and two motors mounted on a linear guide control the racket's position. Based on this platform, researchers from Miyazaki Laboratory proposed a table tennis racket motion planning method based on the mirror image method. They proposed a local weighted regression racket motion planning method to control table tennis's drop point successfully.

In 2007, TOSY of Vietnam and Quanta-view of Japan had successively developed table tennis robots that can play against people. The TOPIO developed by the Vietnam TOSY company uses a binocular camera system to obtain the flight trajectory of table tennis. The third-generation table tennis robot was created in 2010. The overview shows that table tennis robots based on deep learning and machine vision have become a development trend [14].

## 3. Methodology

In this paper, the table tennis ball's precise rotation is reversed through various information such as motion trajectory, speed, and landing point. Since no scholar has studied the relationship between the accurate rotation of table tennis and its trajectory, speed, and drop point before, the premise of reversing the rotation is to prove a correlation between this information. This paper is mainly based on the neural network design algorithm of machine vision and calculates the correlation between table tennis rotation and movement trajectory. This paper will design experiments to obtain accurate initial position coordinates, accurate initial speed size and direction, and accurate rotation speed size and direction. These 9 initial data are used as the input information of the neural network [15, 16], and the precise landing coordinates are used as the output information. Using machine vision algorithms [17, 18], we explore the correlation between input and output information, provide a theoretical and experimental basis for reversing accurate rotation, and make efforts for the subsequent application of table tennis robots to hit rotating balls.

### 3.1. Improved SCG Neural Network Algorithm

The full name of the SCG algorithm is called the scaling conjugate gradient method, which is an improvement based on the conjugate gradient method. The conjugate gradient method is an unconstrained optimization method. Its essence is to improve the direction search of the gradient descent method. The gradient of the previous point is multiplied by an appropriate coefficient and added to the point's speed to obtain a new search direction. Compared with the gradient descent method, the conjugate gradient method mainly solves the shortcomings of slow convergence speed and complicated calculation. It first searches along the direction of the negative gradient and then searches along the current search's conjugate direction, which can shorten the calculation time and reach the optimal value as soon as possible. This method has better applicability for networks with many weights. It has a small amount of data storage and calculation. It has a much faster convergence rate than the conventional gradient descent method. Next, briefly introduce the principle of the conjugate gradient method. Set the connection weight space between the forward BP network's neuron nodes as W, which is an asymmetric matrix with zero elements on the diagonal. The search direction in the basic BP algorithm is *E*, t represents the number of iterations, so adjacent search directions are orthogonally conjugated.

Take the direction of the first step search as the negative gradient direction, then

(1) $$\begin{array}{c} d^{\left(1\right)}=-\frac{\partial E^{\left(0\right)}}{\partial W}. \end{array}$$

Then there are

(2) $$\begin{array}{c} \Delta W\left(1\right)=\lambda d^{\left(1\right)}=-\lambda \frac{\partial E^{\left(0\right)}}{\partial W}, \end{array}$$

where *λ* represents the learning rate, and (2) represents the negative gradient direction of the objective function *E* to the weight space *W* after the first iteration is −*λ*∂*E*^(0)^/∂*W*. According to this method, the downward iteration is performed to construct a new round of iteration parameters as follows:

(3) $$\begin{array}{c} d^{\left(2\right)}=-\lambda \frac{\partial E^{\left(1\right)}}{\partial W}+\beta \Delta W\left(1\right), \end{array}$$

where *β* represents the conjugate factor, which can ensure that *d*^(1)^ and *d*^(2)^ have conjugate properties. According to this iterative method, the search direction of the *t*+1th time can be obtained as

(4) $$\begin{array}{c} d^{\left(t+1\right)}=-\lambda \frac{\partial E^{\left(t\right)}}{\partial W}+\beta^{\left(t\right)}\Delta W\left(1\right). \end{array}$$

According to the above equation, the BP algorithm weight correction formula based on conjugate direction correction is

(5) $$\begin{array}{c} \Delta W\left(t+1\right)=\lambda \left(-\frac{\partial E^{\left(t\right)}}{\partial W}+\beta \Delta W\left(t\right)\right). \end{array}$$

Assuming that the gradient of the objective function *E* in the weight space *W* is ∂*E*^(*t* − 1)^/∂*W* before the *t*th correction, then the *t*th correction calculation can get the gradient of *E* to *W* as ∂*E*^(*t*)^/∂*W*, and the conjugate factor is

(6) $$\begin{array}{c} \beta \left(t\right)=\frac{{\left\|\partial E^{\left(t\right)}|/|\partial W\right\|}^{2}}{{\left\|\partial E^{\left(t-1\right)}|/|\partial W\right\|}^{2}}. \end{array}$$

To ensure the search direction's conjugacy, the initial search direction takes the negative gradient direction; that is, let *β*^(0)^=0, and formulate rules. If the search direction changes to a nondeclining direction due to the accumulation of errors in multiple steps during the search process, restart the correct direction and continue to restart the subsequent search work in the negative gradient direction.

The specific calculation steps are as follows:

1. Select the initial weight *ω*_1_
2. Find the gradient *g*_1_=∇*E|ω*_1_, and the initial search direction is *d*_1_=−*g*_1_
3. In step *j*, adjust the value of *a* so that *E*(*ω*_*j*_+*ad*_*j*_) reaches the minimum value, and continue to calculate the weight *ω*_*j*+1_=*ω*_*j*_+*a*_min_*d*_*j*_ of the next step
4. Check whether the conditions for stopping are met
5. Calculate the new gradient value *g*_*j*+1_
6. Calculate the new search direction according to (6)
7. Let *j*=*j*+1, and return to step 3

In the entire iteration process, the search direction may no longer have conjugate due to the accumulation of errors. The search direction can be reset to the negative gradient direction after running some iterations each time, which can solve the conjugacy problem to a certain extent.

### 3.2. Table Tennis Tracking Based on Machine Vision

In this section, we discuss the proposed algorithm's components to track the tennis ball using machine vision.

#### 3.2.1. Image Segmentation Based on VOCUS System

The VOCUS system is a new type of image segmentation system based on visual attention. The eye gaze model is added to the visual system to achieve effective segmentation of image scenes. Some scholars have discovered that there are three opposing color channels in the human visual system: black and white, red and green, and blue and yellow, and humans can observe the scene through these three color channels. The VOCUS system applies this theory to the system, divides a picture into these three color channel recognitions, and realizes the image segmentation through filtering, difference, normalization, fusion, and other operations. The specific flowchart is shown in Figure 2.

Figure 2 shows the process of image segmentation, and the specific steps are as follows.

1. Step 1: after inputting a picture, use the color information as a linear filter to decompose the input picture into pictures of three channels. The channels are black/white, red/green, and blue/yellow, and the filter thresholds are

(7) $$\begin{array}{c} \text{BW}=\frac{R+G+B}{3},\\ \text{RG}=R-G,\\ \text{BY}=B-Y. \end{array}$$

(2) Step 2: use the image Gaussian pyramid algorithm to blur the image multiple times and downsample to generate multiple sets of images at different scales. This experiment uses 5 sets of pyramid scale images.
(3) Step 3: perform central-peripheral difference and normalization processing on each group of images in turn to generate different feature maps under the three channels. The difference mainly uses the DoG filtering algorithm.
(4) Step 4: perform multiscale feature fusion operation on the feature maps under the three channels to generate a set of prominent images.
(5) Step 5: linearly merge the salient images under the three channels to generate a salient image and realize image segmentation.
(6) Step 6: after the image segmentation is completed, mark the most significant 3 areas with red boxes to facilitate subsequent processing.

#### 3.2.2. Table Tennis Recognition Based on High-Speed Photography

After preprocessing the image, the segmented image can be recognized. This section first recognizes the image under high-speed photography. The selected high-speed camera is placed next to the ping-pong table's sideline, and the speed is 250 frames per second. The shutter selects 1/2000 second to take a picture of the entire trajectory of the ping-pong ball. Because the shooting speed is fast enough and the shutter is high enough, the ping-pong ball shot is clearer, as shown in Figure 3.

As can be easily seen from Figure 4, the image is segmented into three protruding areas, which contain the area where the ping pong ball is located. Next, the three protruding areas will be processed directly to identify the ping pong ball. Since table tennis characteristics are still more obvious after preprocessing, the characteristic information of the table tennis can be used to identify the table tennis.

It can be found from Table 1 that if the detection value of the object is within the set threshold, the object will be recognized as the ping pong ball that needs to be identified. The threshold setting is determined according to the experimental value. After identifying the ping-pong ball area, remove the three red boxes and directly enclose the ping-pong ball with the red box to complete the identification and tracking of the ping-pong ball. The recognition result is shown in Figure 5.

## 4. Experiments

In this section, the details about experiments are discussed in detail. The experimental environments, datasets, and experimental results are elaborated.

### 4.1. Experimental Environment

Table 2 shows the experimental environment of this paper. The systems hardware environment in the experiment is CPU Intel Core i7-4700MQ, 2.4GHZ, 8 GB of memory, and the development platform is MATLAB R2013b with Windows 7 operating system.

### 4.2. Dataset

The experimental data are shown in Table 3. The results shown in this article are all actual data from table tennis robots playing against people. There are a total of 75 sets of valid data. 70 sets of data are used as training samples for the ELM model, and 5 sets of data are used as comparison data.

### 4.3. Experimental Results

Table 4 shows 5 sets of predicted data and actual measured coordinates and their deviation values. It can be seen from Table 4 that the prediction results of the algorithm in this paper show that it is less than 20 mm in the *x*-direction, less than 10 mm in the *y*-direction, and less than 10 mm in the *z*-direction. Aiming at the result of a large amount of data leading to a long training time, this paper adopts saving the network for the next prediction. After getting the expected result, save the network so that the predicted result will not change, and call the network the next time there is new data for prediction.

From Table 5, we can see the maximum error of BP on the *X*-axis, which is 17.5 mm. The proposed algorithm results in 29.2 mm; the maximum error of BP on the *Y*-axis is 5.4 mm. The proposed algorithm is 4.7 mm; the maximum error of BP on the *Z*-axis is 6.5, while the algorithm in this paper is 4.3 mm. After calculation, the mean square error of the three-axis error of the neural network in this paper is 4.663, while the mean square error of the BP algorithm is 9.226. The data shows that the BP algorithm's error is larger than our range, and the fluctuation is also large. Therefore, this proves the effectiveness and superiority of the algorithm in this paper.

## 5. Conclusion

This paper proposes a table tennis target trajectory tracking algorithm based on machine vision combined with SCG. First, obtain real human-machine battle data, extract 10 continuous position information and speed information frames to select features, use them as input data for the deep neural network, and then normalize them to create a deep neural network algorithm model and then output the result. It is the position information of the next 20 frames. Through many experiments, we found the shortcomings of the original SCG algorithm. By setting the accuracy threshold and offline learning of historical data and saving the hidden layer weight matrix, the SCG algorithm was improved to save the trained model. Finally, experiments verify the feasibility and applicability of the improved algorithm. The experimental results also show our algorithm's effectiveness and superiority, which is more suitable for table tennis robots.

## Figures and Tables

**Figure 1:** Ping pong table for the table tennis.

**Figure 2:** Image segmentation flowchart.

**Figure 3:** High-speed camera to take pictures.

**Figure 4:** Image segmentation result.

**Figure 5:** Table tennis recognition result.

**Table 1:** Five characteristics of table tennis.

Type	Description
Roundness	*M*=4*πA*/*C*^2^
Perimeter	The perimeter value of the measurement object, denoted by C
Area	The perimeter value of the measurement object, denoted by A
X distance	The maximum distance value of the measurement object in the horizontal direction, that is, the *X*-axis direction, expressed by Lx2
Y distance	Measure the vertical direction of the object, that is, the maximum distance value in the *Y*-axis direction, expressed in Ly

**Table 2:** Experimental hardware platform and software simulation environment.

CPU	Intel core i7-4700MQ @ 2.40 GHz
RAM	8.00 GB
Operating system	Windows 7
Development environment	MATLAB R2013b

**Table 3:** Examples of datasets.

Index	Measured (*x*, *y*, *z*) (mm)
1	(483.4, 103.6, 272.2)
2	(490.4, 112.1, 280.7)
3	(516.0, 114.1, 292.5)
4	(531.5, 111.9, 301.4)
5	(565.8, 120.2, 315.5)
6	(588.4, 123.0, 325.1)
7	(615.6, 124.1, 335.5)
8	(688.7, 134.3, 356.9)
9	(736.4, 138.6, 367.8)
10	(763.6, 138.3, 368.1)
11	(799.8, 144.9, 373.0)
12	(825.7, 148.2, 373.9)
13	(847.2, 149.6, 373.3)
14	(866.7, 1 S 1.8, 371.0)
15	(896.0, 157.0, 372.7)
16	(920.1, 159.2, 369.7)
17	(940.3, 159.5, 365.4)
18	(956.9, 161.3, 357.8)
19	(978.8, 162.5, 353.4)
20	(1011.0, 170.2, 349.8)

**Table 4:** Experimental results.

Index	Measured (*x*, *y*, *z*) (mm)	Predicted (*x*, *y*, *z*) (mm)	Errors (mm)
1	(483.4, 103.6, 272.2)	(465.9, 109.0, 265.7)	(17.5, -5.4,6.5)
2	(490.4, 112.1, 280.7)	(490.3, 108.0, 280.4)	(0.1, 4.0, 0.2)
3	(516.0, 114.1, 292.5)	(522.2, 114.2, 294.8)	(-6.2, 0.0, -2.3)
4	(531.5, 111.9, 301.4)	(541.5, 115.5, 301.2)	(-10.0, -3.5, 0.2)
5	(1011.0, 170.2, 349.8)	(1005.7, 169.8, 348.7)	(5.3, 0.4, 1 .1)

**Table 5:** Comparison of experimental results.

Index	Ours	BP neural network
1	(17.5, −5.4,6.5)	(4.1, −3.1, −4.2)
2	(0.1,4.0,0.2)	(−24.2, 3.7, 0)
3	(−6.2,0.0,−2.3)	(7.8, −3.6, 0.5)
4	(−10.0,−3.5,0.2)	(10, −3.9, −5)
5	(5.3,0.4,1 .1)	(−18, 4.6, −2.6)

## Data Availability

The data used to support the findings of this study are included within the article.
